The article "Efficacy of Qingfei Paidu Decoction on Patients with COVID-19 Pneumonia in Wuhan, China: A Propensity Score Matching Study" was published in 2021. Journal: Evid Based Complement Alternat Med.

# Efficacy of Qingfei Paidu Decoction on Patients with COVID-19 Pneumonia in Wuhan, China: A Propensity Score Matching Study

**DOI:** 10.1155/2021/4303380

**Published:** 2021-10-05

**Authors:** Zhen Liu, Shan Du, Fei Shao, Haibin Li, Shuang Xu, Xuedi Ma, Zhouming Xu, Hao Cui, Changxiao Yu, Yang Wu, Feng Wang, Liyan Li, Rui Chen, Hui Qiu, Ziren Tang, Peng Sun

**Affiliations:** ^1^Department of Emergency Medicine, Beijing First Hospital of Integrated Chinese and Western Medicine, Beijing, China; ^2^Department of Neurology, Beijing First Hospital of Integrated Chinese and Western Medicine, Beijing, China; ^3^Department of Emergency Medicine, Beijing Chaoyang Hospital, Capital Medical University, Beijing, China; ^4^Beijing Key Laboratory of Cardiopulmonary Cerebral Resuscitation, Beijing, China; ^5^Department of Epidemiology and Health Statistics, School of Public Health, Capital Medical University, Beijing, China; ^6^Department of Emergency Medicine, Union Hospital, Tongji Medical College, Huazhong University of Science and Technology, Wuhan, China; ^7^AI Research Division, A.I. Phoenix Technology Co., Ltd., Hong Kong, China; ^8^Department of Respiratory and Critical Care Medicine, Beijing Chaoyang Hospital, Capital Medical University, Beijing, China; ^9^Beijing Key Laboratory of Respiratory and Pulmonary Circulation Disorders, Beijing, China; ^10^Department of Integrated Traditional Chinese and Western Medicine, Union Hospital, Tongji Medical College, Huazhong University of Science and Technology, China; ^11^Department of Emergency Surgery, the West Campus of Union Hospital, Tongji Medical College, Huazhong University of Science and Technology, Wuhan, China

## Abstract

**Background:**

In view of the global efforts to develop effective treatments for the current worldwide coronavirus 2019 (COVID-19) pandemic, Qingfei Paidu decoction (QPD), a novel traditional Chinese medicine (TCM) prescription, was formulated as an optimized combination of constituents of classic prescriptions used to treat numerous febrile and respiratory-related diseases. This prescription has been used to treat patients with COVID-19 pneumonia in Wuhan, China. *Hypothesis/Purpose*. We hypothesized that QPD would have beneficial effects on patients with COVID-19. We aimed to prove this hypothesis by evaluating the efficacy of QPD in patients with COVID-19 pneumonia.

**Methods:**

In this single-center, retrospective, observational study, we identified eligible participants who received a laboratory diagnosis of COVID-19 between January 15 and March 15, 2020, in the west campus of Union Hospital in Wuhan, China. QPD was supplied as an oral liquid packaged in 200-mL containers, and patients were orally administered one package twice daily 40 minutes after a meal. The primary outcome was death, which was compared between patients who did and did not receive QPD (QPD and NoQPD groups, respectively). Propensity score matching (PSM) was used to identify cohorts.

The article "Efficacy of Qingfei Paidu Decoction on Patients with COVID-19 Pneumonia in Wuhan, China: A Propensity Score Matching Study" was published in 2021. Journal: Evid Based Complement Alternat Med.

**Results:**

In total, 239 and 522 participants were enrolled in the QPD and NoQPD groups, respectively. After PSM at a 1 : 1 ratio, 446 patients meeting the criteria were included in the analysis with 223 in each arm. In the QPD and NoQPD groups, 7 (3.2%) and 29 (13.0%) patients died, and those in the QPD group had a significantly lower risk of death (hazard ratio (HR) 0.29, 95% CI: 0.13–0.67) than those in the NoQPD group (*p* = 0.004). Furthermore, the survival time was significantly longer in the QPD group than in the NoQPD group (*p* < 0.001).

**Conclusion:**

The use of QPD may reduce the risk of death in patients with COVID-19 pneumonia.

## 1. Introduction

The outbreak of the novel coronavirus pandemic has affected more than 200 countries globally, and as of March 1, 2021, over 113,467,303 confirmed cases of coronavirus disease 2019 (COVID-19) have been reported with over 2,520,550 deaths [1]. The novel coronavirus was identified as severe acute respiratory syndrome coronavirus 2 (SARS-CoV-2), and the associated disease COVID-19 has clinical manifestations ranging from asymptomatic, mild pneumonia to serious acute respiratory distress syndrome, septic shock, and multiple organ dysfunction syndrome (MODS) [2–4].

Currently, despite supportive and symptomatic treatments, no specific medicine is recommended for the prevention or treatment of COVID-19 and many countries and organizations are racing against time to identify prophylactic and therapeutic treatments for patients [5]. On January 26, 2020, a new TCM prescription named Qingfei Paidu decoction (QPD) was formulated with expert consensus using a combination of 21 traditional Chinese medicine (TCM) ingredients based on previous clinical experience and disease data [6].

After the National Health Commission of the People's Republic of China (NHCPRC) released the QPD Diagnosis and Treatment Protocol for Novel Coronavirus Pneumonia (Trial Version 6) on February 19, 2020 [7], QPD was widely administered for the treatment of patients with COVID-19 nationally in China. Therefore, we aimed to explore the effects of QPD in patients with COVID-19 pneumonia.

## 2. Methods

### 2.1. Study Design

This was a single-center, retrospective, observational study comparing the clinical effectiveness of a combination of QPD and standard therapy versus standard therapy alone in the treatment of patients with COVID-19 pneumonia. The study was approved by the Ethics Committee Boards of Union Hospital, Tongji Medical College, and Huazhong University of Science and Technology, and the requirement for informed consent was waived on account of the retrospective study design.

The article "Efficacy of Qingfei Paidu Decoction on Patients with COVID-19 Pneumonia in Wuhan, China: A Propensity Score Matching Study" was published in 2021. Journal: Evid Based Complement Alternat Med.

### 2.2. Study Population and Setting

We identified patients who received a laboratory diagnosis of COVID-19 between January 15 and March 15, 2020, at the west campus of Union Hospital in Wuhan. The eligibility criteria were as follows: aged ≥14 years and diagnosed with COVID-19 according to the interim guidelines of the World Health Organization. All enrolled inpatients had a definite outcome and received in-hospital care consistent with the Diagnosis and Treatment Protocol for Novel Coronavirus Pneumonia (Trial Version 6) recommended by the NHCPRC [7].

The west campus of Union Hospital was one of the designated hospitals for patients with severe COVID-19, and 800 beds were modified as isolation wards and opened for admission to patients from January 2020. The Department of TCM was in charge of evaluating the clinical needs of patients and prescribing TCM drugs according to their symptoms and clinical features. The TCM pharmacy was provided QPD prescriptions, which were used to produce a decoction for patients in the general ward or intensive care unit (ICU).

### 2.3. QPD Exposure

According to the Diagnosis and Treatment Protocol for Novel Coronavirus Pneumonia (Trial Version 6) of the NHCPRC, patients with COVID-19 were cotreated with QPD and standard agents [7]. All patients in the general ward or ICU were administered QPD with the combination of Western medicine from the first day after hospital admission. Patients who met the following exclusion criteria were excluded: gastrointestinal bleeding before use of QPD, refused to take QPD, or coma patients without a feeding tube. Physicians of the Department of TCM evaluated the clinical features of the patients and prescribed QPD to those in the general ward or ICU.

The QPD was formulated as an oral liquid with each package containing 200 mL. The patients received one package of QPD twice a day, in the morning and evening, 40 minutes after a meal. Patients with dry tongue due to fluid depletion were recommended to consume one bowl of rice soup. The amount of gypsum should be increased for patients with moderate or high fever. A treatment course was considered to be 3 days and was followed by another course of QPD if the symptoms improved but the patient had not totally recovered.

Patients with specific or other underlying diseases could be administered formulas in the subsequent course that were modified according to their actual conditions. QPD treatment was discontinued if the patient's symptoms were resolved, effects associated with contraindicated oral administration were observed, or severe adverse effects related to QPD occurred [7].

The article "Efficacy of Qingfei Paidu Decoction on Patients with COVID-19 Pneumonia in Wuhan, China: A Propensity Score Matching Study" was published in 2021. Journal: Evid Based Complement Alternat Med.

### 2.4. Data Collection

Information on age, sex, clinical symptoms, treatments, comorbidity, and outcome data of patients with severe COVID-19 pneumonia treated with QPD was retrieved from their electronic medical records by the physicians and entered into a database during the study period. The primary outcome was death before discharge from hospital.

### 2.5. Statistical Analysis

Nominal data are described using proportions, normally distributed discrete data are described as means and standard deviation (SD), and medians and interquartile ranges (IQRs) are used to represent data that were not normally distributed. Because the baseline characteristics of eligible participants differed between the two groups (Table 1), propensity score matching (PSM) was used to identify a cohort of patients with similar baseline characteristics. The propensity score was set as a conditional probability of having a particular exposure (QPD versus NoQPD) considering a set of baseline measured covariates.

The propensity score was estimated using a nonparsimonious multivariable logistic regression model with QPD as the dependent variable and all baseline characteristics outlined in Table 1 as covariates. Matching was performed using a 1 : 1 matching protocol without replacement (greedy matching algorithm) with caliper width = 0.2 times the SD of the propensity score logit. Absolute standardized mean differences of less than 10.0% for a given covariate indicate a relatively small imbalance.

Patient data were analyzed from baseline to the date of death or discharge, and the primary outcome was based on the PSM. Kaplan–Meier survival curves and stratified log-rank tests were used, and the hazard ratio (HR) and corresponding 95% confidence intervals (CIs) were calculated using the Cox proportional hazard models.

Analyses were performed using R version 3.6.3, all tests were two-sided, and *p* values < 0.05 were considered statistically significant.

## 3. Results

From January 15 to March 15, 2020, 792 inpatients with COVID-19 were assessed for eligibility. Thirty-one patients were excluded, with 4 not meeting the inclusion criteria and 27 missing data (Figure 1). In total, we identified 761 eligible participants, comprising 239 and 522 who were treated with and without QPD, respectively, and the patient characteristics are shown in Table 1. In the unmatched comparison of baseline characteristics of patients, no differences were observed between the QPD and NoQPD groups in sex and age. Among the variables analyzed, symptoms of nausea, myalgia, mental abnormalities, and diabetes as a comorbidity were significantly different between the two groups (Table 1).

The article "Efficacy of Qingfei Paidu Decoction on Patients with COVID-19 Pneumonia in Wuhan, China: A Propensity Score Matching Study" was published in 2021. Journal: Evid Based Complement Alternat Med.

After PSM at a 1 : 1 ratio, 446 patients meeting the criteria were included in the analysis with 223 patients in each arm. The mean age of the QPD and NoQPD groups was 59 and 61 years, and 50.2% and 49.3% of the participants were women, respectively (Table 2). Baseline demographic characteristics, symptoms, and comorbidities were almost comparable between the two groups except for the history of diabetes (Table 2). Furthermore, 7 (3.2%) and 29 (13.0%) patients died in the QPD and NoQPD groups, respectively.

Patients in the QPD group had a significantly (*p* = 0.004) lower risk of death (HR 0.29, 95% CI: 0.13–0.67) than those in the NoQPD group. We also conducted a sensitivity analysis, and after adjusting for baseline age, sex, and diabetes, patients in the QPD group also showed a significantly (*p* = 0.004) lower risk of death (HR 0.30, 95% CI: 0.13–0.68) than those in the NoQPD group (Table 3).  Figure 2 shows the Kaplan–Meier survival curves.

## 4. Discussion

This retrospective analysis showed that cotreatment of patients with COVID-19 pneumonia with QPD and conventional treatment was associated with higher rates of survival and hospital discharge, lower death rates, and longer survival time than conventional treatment alone. Following the outbreak of COVID-19, timely intervention using TCM has played an important role in its treatment in China. The NHCPRC issued seven versions of its diagnosis and treatment protocol for COVID-19 with recommendations to combine TCM prescriptions and standard treatment since the third version was issued on January 23, 2020 [7–9].

TCM is a complete theoretical system that has played an indispensable role in the prevention and treatment of several epidemic diseases in China over the years [10]. For instance, in 2003, TCM prescriptions were used to prevent and treat SARS. TCM herbal extracts of *Cibotium barometz*, *Gentiana scabra*, *Dioscorea batatas*, *Cassia tora*, and *Taxillus chinensis* can inhibit SARS-CoV replication [11]. During the influenza A virus subtype H1N1 (H1N1) influenza pandemic of 2009, oseltamivir and maxingshigan-yinqiaosan alone and in combination with standard agents reduced time to fever resolution in infected patients. Consequently, maxingshigan-yinqiaosan may be an alternative treatment for H1N1 influenza virus infection [12].

QPD is an optimized combination of classic prescriptions used for the treatment of multiple exogenous febrile diseases. It is composed of 21 herbs (Table 4) derived from Maxing Shigan decoction (MSD), Shegan Mahuang decoction (SMD), Xiaochaihu decoction (XCHD), and Wuling powder in the “Treatise on Febrile and Miscellaneous Diseases” by Dr. Zhang Zhongjing in the Han Dynasty. Among these constituents, the main active ingredient is MSD, which consists of Herba Ephedrae, Semen armeniacae amarum, Gypsum fibrosum, and Radix Glycyrrhizae.

The article "Efficacy of Qingfei Paidu Decoction on Patients with COVID-19 Pneumonia in Wuhan, China: A Propensity Score Matching Study" was published in 2021. Journal: Evid Based Complement Alternat Med.

MSD has been widely used in the prevention and treatment of respiratory diseases. Several studies had verified its antiviral effects mediated by regulating immune function, suppressing inflammatory cytokine storm, and improving oxygenation and forced expiratory volume/second (FEV1) [13, 14]. SMD has been shown to alleviate pathological lung damage and inflammation in rats with asthmatic pneumonia by enhancing immune activity and downregulating the expression of thymic stromal lymphopoietin (TSLP), toll-like receptor 4 (TLR4), and nuclear factor-*κ*B (NF-*κ*B) in lung tissue [15].

XCHD has immunomodulatory, anti-liver injury, and anti-inflammatory effects mediated by regulating the level of pathogens on the half-superficies and half-interior and inhibiting the inflammatory cytokines tumor necrosis factor (TNF-*α*), IL-1*β*, IL-6, and macrophage colony-stimulating factor (M-CSF) [16, 17]. Wuling powder possesses strong anti-inflammatory activity and acts through various signaling pathways, including NF-*κ*B, mitogen-activated protein kinases (MAPKs), and heme oxygenase-1 (HO-1) [18].

A pharmacokinetic study has shown that the potent inhibition of CYP1A and CYP3A by QPD partially blocks the formation of the oxidative metabolites of arachidonic acid, thereby alleviating systemic inflammation in patients with COVID-19. Thus, QPD may exert its anti-inflammatory effects by inhibiting human P450s [19]. Some core components of QPD have an affinity for the novel SARS-CoV-2 main protease (3C-like protease, 3CLpro) and angiotensin-converting enzyme 2 (ACE2) [20]. Furthermore, by regulating a series of proteins coexpressed with ACE2 and signaling pathways closely related to the occurrence and development of diseases, it plays a role in balancing immunity and eliminating inflammation. It may act as an antiviral agent by targeting ribosomal proteins that are necessary for viral replication, thereby inhibiting viral mRNA translation and a group of proteins that interact with viral proteins [21].

As indicated in the sixth edition of the recommendation guidelines, QPD is suitable for mild, moderate, and severe cases of COVID-19 in accordance with clinical observations of doctors in various locations and can be used reasonably after considering the actual conditions of critically ill patients [7]. Under the guidance, patients should be administered QPD with appropriately adjusted constituents according to their specific conditions, such as body temperature, diet, and symptoms.

The article "Efficacy of Qingfei Paidu Decoction on Patients with COVID-19 Pneumonia in Wuhan, China: A Propensity Score Matching Study" was published in 2021. Journal: Evid Based Complement Alternat Med.

Studies have shown that the combination of QPD and conventional treatment relieves the symptoms of COVID-19 and resolves inflammation in the lung [22]. Early treatment with QPD may serve as an effective strategy in controlling the pandemic, as early treatment with QPD is associated with favorable outcomes, including faster recovery, shorter time to viral shedding, and shorter duration of hospital stay [23]. Although the mechanism of the pharmacological action of QPD in the treatment of COVID-19 is complex, its primary site of action is the lung, which indicates that the decoction has specific effects against lung diseases [24]. Moreover, two studies with small samples have suggested that QPD combined with Western medicine in the treatment of COVID-19 is more effective than western medicine alone and can significantly shorten the patient's hospitalization time, clinical symptom improvement time, and lung CT improvement time; however, neither mortality nor length of hospitalization was affected [25].

QPD includes ephedra, which is banned in the US due to toxicity and is not considered safe by the EFSA. The ban on ephedra-containing supplements continues to be controversial. Ephedra is legal and widely used in several countries, such as Germany, Japan, India, and China. According to the Chinese Pharmacopoeia, Herba Ephedrae (ma huang) has a total alkaloid content of 1% by dry weight, and honey-frying decreases the alkaloid content by 0.194%. The safe daily dose of Herba Ephedrae is 2–9 g/d. QPD contains 9 g of Herba Ephedrae and caused no serious adverse effects.

Our study found that the administration of QPD reduced the mortality rate of patients with COVID-19 and for the British and Indian COVID-19 variants that are currently emerging, Traditional Chinese medicine may be an option. In the future, high-quality, prospective, controlled studies are required to confirm the efficacy and the safety; meanwhile, basic research is also needed to explore the mechanisms of TCM prescriptions to provide new approaches for the treatment of COVID-19.

### 4.1. Limitations

Notably, there are some limitations to this study. First, although we used PSM to eliminate the bias caused by confounders, unmeasured and residual confounding factors could still have influenced our results. For example, the timing of administration and sequence in relation to other interventions, severity of illness among patients, or a combination of these factors may have differed between those treated with and without QPD. Second, some risk factors, such as D-dimer, sequential organ failure assessment score, and lactate dehydrogenase [4, 26], were not included in our analysis. Third, there are few pharmacokinetic studies on QPD because it is a new formulation developed during the recent COVID-19 outbreak. Further studies to explore the mechanisms of action of QPD are needed. Lastly, other TCM formulations were administered to patients in the study and we could not specify their effects, which could have affected the result of this study.

The article "Efficacy of Qingfei Paidu Decoction on Patients with COVID-19 Pneumonia in Wuhan, China: A Propensity Score Matching Study" was published in 2021. Journal: Evid Based Complement Alternat Med.

## 5. Conclusions

QPD may reduce the risk of death in patients with COVID-19. Further randomized controlled clinical trials are needed to corroborate these findings and provide definite conclusions. Finally, pharmacokinetic studies on QPD and its expanded use are needed in the future.

## Figures and Tables

**Figure 1:** Flow diagram illustrating the number of patients during the study.

**Figure 2:** Survival curve by treatment group.

**Table 1:** Characteristics of patients with COVID-19 pneumonia.

Variables	QPD	NoQPD	SMD
*n*	239	522	

*Sex*			
Female (%)	120 (50.2)	251 (48.1)	0.043

*Age* (median [IQR])	60.00 [51.00–66.00]	62.00 [50.00–70.00]	0.022

*Symptoms*			
Fever	192 (80.3)	439 (84.1)	0.099
Dizziness	27 (11.3)	51 (9.8)	0.050
Fatigue	128 (53.6)	278 (53.3)	0.006
Nausea	35 (14.6)	51 (9.8)	0.149
Diarrhea	46 (19.2)	100 (19.2)	0.002
Myalgia	62 (25.9)	111 (21.3)	0.110
Abnormality of mentality	9 (3.8)	72 (13.8)	0.360
Headache	18 (7.5)	26 (5.0)	0.105
Abdominal pain	13 (5.4)	20 (3.8)	0.077
Dyspnea	179 (74.9)	367 (70.3)	0.103
Cough	188 (78.7)	395 (75.7)	0.071
Sputum	105 (43.9)	214 (41.0)	0.059
Chest pain	14 (5.9)	22 (4.2)	0.075

*Comorbidity*			
Hypertension	45 (18.8)	105 (20.1)	0.032
Diabetes	21 (8.8)	18 (3.4)	0.224
Coronary heart disease	13 (5.4)	36 (6.9)	0.061
COPD	1 (0.4)	3 (0.6)	0.022
Cancer	6 (2.5)	14 (2.7)	0.011
Chronic renal disease	0 (0.0)	2 (0.4)	0.088
Cerebrovascular disease	5 (2.1)	12 (2.3)	0.014

SMD >0.1 indicates a difference in baseline characteristics between both groups. QPD, Qingfei Paidu decoction; SMD, standardized mean difference; IQR, interquartile range; COPD, chronic obstructive pulmonary disease.

**Table 2:** Characteristics of patients with COVID-19 pneumonia after propensity score matching (1 : 1 match).

Variables	QPD	NoQPD	SMD
*n*	223	223	

*Sex*			
Female (%)	112 (50.2)	110 (49.3)	0.018

*Age* (median [IQR])	59.00 [51.00–66.00]	61.00 [49.00–69.00]	0.001

*Symptoms*			
Fever	179 (80.3)	184 (82.5)	0.058
Dizziness	24 (10.8)	25 (11.2)	0.014
Fatigue	119 (53.4)	121 (54.3)	0.018
Nausea	33 (14.8)	35 (15.7)	0.025
Diarrhea	43 (19.3)	45 (20.2)	0.023
Myalgia	56 (25.1)	62 (27.8)	0.061
Abnormality of mentality	9 (4.0)	8 (3.6)	0.023
Headache	18 (8.1)	15 (6.7)	0.051
Abdominal pain	13 (5.8)	12 (5.4)	0.019
Dyspnea	164 (73.5)	164 (73.5)	<0.001
Cough	174 (78.0)	169 (75.8)	0.053
Sputum	100 (44.8)	90 (40.4)	0.091
Chest pain	14 (6.3)	10 (4.5)	0.080

*Comorbidity*			
Hypertension	43 (19.3)	39 (17.5)	0.046
Diabetes	17 (7.6)	10 (4.5)	0.132
Coronary heart disease	11 (4.9)	14 (6.3)	0.059
COPD	1 (0.4)	1 (0.4)	<0.001
Cancer	6 (2.7)	6 (2.7)	<0.001
Chronic renal disease	0 (0.0)	0 (0.0)	<0.001
Cerebrovascular disease	5 (2.2)	5 (2.2)	<0.001

QPD, Qingfei Paidu decoction; SMD, standardized mean difference; IQR, interquartile range; COPD, chronic obstructive pulmonary disease. All variables except diabetes had SMD values less than 0.1, indicating that the two groups were comparable.

The article "Efficacy of Qingfei Paidu Decoction on Patients with COVID-19 Pneumonia in Wuhan, China: A Propensity Score Matching Study" was published in 2021. Journal: Evid Based Complement Alternat Med.

**Table 3:** Outcome event analysis of samples based on propensity score matching.

	Death rate	HR (95% CI)^*∗*^	*p* value	HR (95% CI)^#^	*p* value
NoQPD (*n* = 223)	29 (13.0%)	1.00		1.00	
QPD (*n* = 223)	7 (3.2%)	0.29 [0.13–0.67]	0.004	0.30 [0.13–0.68]	0.004

QPD, Qingfei Paidu decoction; HR, hazard ratio. ^*∗*^Unadjusted. ^#^Adjusted for baseline age, sex, and diabetes.

**Table 4:** Ingredient list of the Qingfei Paidu decoction.

	Ingredients in Chinese	Ingredients in English	Ingredients in Latin	Dose (g)
1	Ma huang	Ephedra herb	Herba ephedrae	9
2	Gan cao, baked	Liquorice root	Radix glycyrrhizae	6
3	Ku xing ren	Bitter apricot seed	Semen armeniacae amarum	9
4	Sheng shi gao	Gypsum	Gypsum fibrosum	15–30
5	Gui zhi	Cassia twig	Ramulus cinmomi	9
6	Ze xie	Oriental waterplantain rhizome	Rhizoma alismatis	9
7	Zhu ling	Agaric	Polyporus umbellatus	9
8	Bai zhu	Largehead atractylodes rhizome	Atractylodis macrocephalae rhizoma	9
9	Fu ling	Tuckahoe	Poria	15
10	Chai hu	Chinese thorowax root	Stellariae radix	16
11	Huang qin	Baical skullcap root	Radix scutellariae	6
12	Jiang ban xia	Ginger processed pinellia	Pinelliae rhizoma praeparatum cum zingibere	9
13	Sheng jiang	Common ginger	Rhizoma zingiberis recens	9
14	Zi wan	Tatarian aster root	Radix asteris	9
15	Kuan dong hua	Common coltsfoot flower	Flos farfarae	9
16	She Gan	Blackberry lily rhizome	Rhizoma belamcandae	9
17	Xi xin	Manchurian wildginger	Herba asari	6
18	Shan yao	Common yam rhizome	Rhizoma dioscoreae	12
19	Zhi shi	Immature bitter orange	Fructus aurantii immaturus	6
20	Chen pi	Tangerine peel	Pericarpium citri reticulatae	6
21	Guang huo xiang	Benth cablin patchouli herb	Pogostemon cablin	9

## Data Availability

The datasets used and/or analyzed during the current study are available from the corresponding author on reasonable request.

## Abbreviations

COVID-19: Coronavirus disease 2019
PSM: Propensity score matching
QPD: Qingfei Paidu decoction
TCM: Traditional Chinese medicine.
